The article "Infertility Due to a Novel Variant of a Balanced Y;1 Translocation: A Case Report" was published in 2025. Journal: Cureus.

# Infertility Due to a Novel Variant of a Balanced Y;1 Translocation: A Case Report

**DOI:** 10.7759/cureus.87327

**Published:** 2025-07-05

**Authors:** Somer Magnuson, Kasey Doney, Logan B Wesemann, Kelli Gross

**Affiliations:** 1 Urology, Rocky Vista University College of Osteopathic Medicine, Ivins, USA; 2 Urology, University of Utah Health, Salt Lake City, USA

**Keywords:** balanced translocation, case report, cryptozoospermia, male factor infertility, testicular sperm aspiration (tesa)

## Abstract

This report describes a 26-year-old male presenting with primary infertility due to severe cryptozoospermia. Diagnostic evaluation revealed a novel balanced translocation at 46,X, t(Y;1)(q11.21,p32.1) and heterozygote carrier status for dysferlinopathy (DYSF). The patient's hormonal profile was normal, and Y chromosome microdeletion testing was negative. Despite testicular sperm aspiration (TESA) and two rounds of in vitro fertilization (IVF) with intracytoplasmic sperm injection (ICSI), fertilization and embryo development were poor. This case highlights the challenges in diagnosing and treating male infertility associated with rare Y;1 translocations and emphasizes the need for further research to improve management strategies.

## Introduction

Infertility is common throughout the world, affecting 15% of couples attempting to conceive. About half of the cases involve male factor infertility [1]. Male infertility can be a multifactorial condition whose etiology is difficult to determine due to the complexity of possible genetic aberrations and the heterogeneous nature of other contributory factors [2]. One such anomaly is a balanced Y;1 translocation, a reciprocal exchange of equal segments between chromosome Y and chromosome 1, without any net loss or gain of genetic material [3]. This type of translocation is exceptionally rare; only a handful of cases have been reported in the literature [3]. The most common manifestations of Y;1 balanced translocations include azoospermia and oligozoospermia, defined as the absence of spermatozoa in the sediment of a centrifuged semen sample and low spermatozoa concentration in a semen sample, respectively [3,4]. Y;1 translocation has also been associated with Hodgkin’s disease [5], spontaneous abortions [6], and craniosynostosis in Y;1 offspring [7]. Most of these cases presented with non-obstructive azoospermia (NOA), a form of azoospermia associated with spermatogenic arrest rather than obstruction of the vas deferens. Current guidelines for the evaluation of male infertility are outlined by the American Urological Association [8]. Initial management of male infertility depends on the results of an initial semen analysis. This evaluation should encompass a physical examination, assessment of semen volume and pH, and hormonal testing (including serum levels of follicle-stimulating hormone (FSH), luteinizing hormone (LH), and testosterone) to distinguish between obstructive and non-obstructive causes of infertility. For azoospermic men, further diagnostic testing, including karyotype analysis and Y-chromosome microdeletion screening, is recommended. Cystic fibrosis transmembrane conductance regulator (CFTR) mutation carrier testing may be considered for cases of vasal agenesis or idiopathic obstructive azoospermia. If a CFTR mutation is detected, evaluation of the partner is advised. Sperm DNA fragmentation and antisperm antibody testing are generally not indicated in the initial work-up unless there is a history of recurrent pregnancy loss. For males with NOA, microsurgical testicular sperm extraction (micro-TESE) should be performed for sperm retrieval; however, conventional testicular sperm extraction (TESE) and testicular sperm aspiration (TESA) are also viable options. Patients should also be made aware of the sparse data supporting the use of pharmacologic manipulation prior to these procedures. In this case, our patient had a semen analysis abnormal for cryptozoospermia, or "hidden sperm," a severe form of oligozoospermia defined by less than 100,000 sperm per milliliter of semen and absence of sperm in microscopic examination but present in centrifuge sediment [8]. The current guidelines show that if no sperm is retrieved following surgical retrieval due to a primary defect, there are no further treatments that can be done for the male [9]. Adding this case to the current literature will provide information on a novel variant of balanced translocations of Y;1 and give another perspective on the difficulties of treating this condition and the struggles affected couples face in cryptozoospermia.

## Case presentation

The 26-year-old male patient presented to the fertility clinic due to primary infertility after one and a half years of trying to conceive with his wife. His 26-year-old wife had been evaluated by a fertility specialist who found no abnormalities. Neither had a prior history of conception. The patient reported no additional complaints or symptoms. He has a fraternal twin brother with a history of varicocele who had not attempted conception, as well as other siblings who were able to conceive without assistance. The patient is a generally healthy male with no significant childhood illnesses that might have impacted fertility. He has no history of chronic medication use and reports no other notable medical conditions. He was able to initiate and maintain an erection and reach ejaculation. His physical exam revealed normal testicular volume, palpable bilateral vas deferens and epididymis, and no varicocele. Hormonal evaluation, including testosterone, FSH, and LH, all of which were within normal limits. Analysis of the microdeletion of the Y chromosome was investigated, and the result was negative. Initial semen analysis (SA) samples showed normal ejaculate volumes but no sperm visible on the initial slide. Following raw sample centrifugation, no sperm were observed on two confirmation slides. The patient was referred for genetic testing to evaluate for potential heritable mutations. He was also advised to return to the clinic for a repeat SA in approximately six to eight weeks. Repeat SA showed similar findings requiring centrifugation, which found one sperm lacking motility. 

As a result of both semen analyses showing very rare sperm after centrifugation, the patient was diagnosed with cryptozoospermia. Karyotype analysis revealed a balanced translocation at 46,X, t(Y;1)(q11.21,p32.1) locus. He was also found to be a heterozygote carrier for dysferlinopathy (DYSF) through genetic carrier panel testing, which has no known clinical significance in male infertility. Consequently, the patient was referred to a genetic counselor who reviewed his diagnosis and discussed the implications. Beyond an acknowledgment that the translocation was contributing to difficulty conceiving, the patient was provided with little detailed information about the exact loci involved. The counselor discussed reproductive options with the couple, including donor sperm, adoption, and in vitro fertilization (IVF) with preimplantation genetic testing for aneuploidy (PGT-A) and structural rearrangements (PGT-SR). They declined the options of using donor sperm and adoption but did agree to IVF with PGT and were referred to appropriate clinics. As shown in Table 1, the patient’s laboratory findings were all within normal range, including hormone levels, and negative for Y-chromosome microdeletion.

**Table 1:** Patient laboratory test results and corresponding reference ranges Reference ranges are based on Labcorp (Labcorp., North Carolina, USA) laboratory test reference ranges [10].

Laboratory Test	Results	Reference Range
Hematocrit (%)	50.9	37.5-51%
Prolactin (ng/mL)	6.9	3.6-31.5
Follicle stimulating hormone (mIU/mL)	10.13	1.5-12.4
Estradiol (pg/mL)	14.27	7.6-42.6
Luteinizing hormone (mIU/mL)	6.55	1.7-8.6
Thyroid stimulating hormone (μIU/mL)	2.953	0.45-4.5
Testosterone, serum (ng/dL)	459	264-916
Sex hormone binding globulin (nmol/L)	31.2	16.5-55.9
Albumin, serum (g/dL)	5.1	4.3-5.2
Y-chromosome microdeletion	Negative	Negative

Due to the patient's consistent cryptozoospermia, he and the urologist decided to proceed with bilateral TESA to cryopreserve sperm with potentially higher counts, along with continued cryopreservation of ejaculated sperm. TESA revealed fibrotic tubules, complicating tissue aspiration, but an adequate sample was obtained, which showed no sperm. Due to the TESA results and discussion with his urologist, the patient opted against further exploring sperm extraction via TESE or micro-TESE due to the financial burden. Subsequently, the couple underwent two rounds of IVF using frozen ejaculated samples. Over several months, the patient provided ejaculate samples for cryopreservation, with the goal of preserving 10 vials of sperm, as agreed upon by the urologist and the patient. Each sample was centrifuged, meticulously examined under more than 200 low-power fields, and thoroughly searched. Samples without sperm were discarded, while those containing a small number of non-motile sperm were preserved.

In both IVF rounds, the patient’s wife responded appropriately to ovarian stimulation. In the first round, 20 oocytes were retrieved, 18 of which displayed adequate maturation (in metaphase II or MII). Ten eggs were injected with frozen sperm, and eight eggs were injected with fresh sperm collected via intracytoplasmic sperm injection (ICSI). All sperm used were immotile and highly amorphous. Successful fertilization was achieved in five of the 18 oocytes injected with frozen sperm, indicating a fertilization rate of 28%. Unfortunately, no embryos progressed to the blastocyst stage suitable for implantation. Six months later, a second round of IVF was performed with similar results. Twenty-one eggs were retrieved, and 14 oocytes showing evidence of nuclear maturation (MII) were injected with sperm via ICSI, which yielded seven successfully fertilized oocytes; however, none progressed to the blastocyst stage. Table 2 provides a detailed sequence of events in the patient's care.

**Table 2:** Timeline of events FSH: follicle-stimulating hormone; LH: luteinizing hormone; TESA: testicular sperm aspiration; ICSI: intracytoplasmic sperm injection; IVF: in vitro fertilization

Event	Details
Presentation to the fertility clinic	A 26-year-old male with primary infertility, 1.5 years trying to conceive. No prior conceptions.
Wife’s evaluation	No abnormalities found in wife’s fertility evaluation.
Family history	Twin with varicocele; siblings are fertile without assistance.
Physical exam	Normal testicular volume, no varicocele.
Hormonal evaluation	Normal testosterone, FSH, and LH levels.
Micro-Y deletion analysis	Negative result.
Semen analysis	Cryptozoospermia diagnosed (<1 million sperm/mL, one motile sperm found).
Genetic testing	Karyotype: balanced translocation at 46,X, t(Y;1)(q11.21,p32.1); DYSF heterozygote carrier.
Genetic counselling	Implications of translocation discussed.
Surgical intervention (TESA)	Bilateral TESA attempted; fibrotic tubules noted; no sperm obtained from testicular tissue.
IVF round 1	20 eggs retrieved, 18 inseminated, five fertilized with ICSI; embryos failed to progress to implantation. Sperm is immotile and amorphous.
IVF round 2	21 eggs retrieved, 14 inseminated, seven fertilized; embryos failed to progress to implantation. Sperm is immotile and amorphous.

## Discussion

The patient’s exact karyotype, 46, X, t(Y;1)(q11.21,p32.1) is a novel variant not previously described in the literature. Similar karyotypes involving balanced reciprocal translocation of chromosomes Y and 1 with similar presentations of male infertility due to azoospermia have been reported [5-7,10,11]. To our knowledge, only 12 other variants of Y;1 translocations have been described in literature, with most cases presenting as azoospermia or oligozoospermia and one case with cryptozoospermia [3,6]. Yq11 has been identified to contain the azoospermia factor (AZF) genes, with q11.21 corresponding to AZFa [12]. Microdeletions of AZF genes have been found to be one of the most common genetic causes of male infertility, indicating that this gene is critical to producing an appropriate number of sperm and may have an effect on its quality [12]. One study showed that individuals with AZFa and AZFb microdeletions had Sertoli cells only with a complete or nearly complete absence of Leydig cells. Microdeletions of AZFa, b, and c genes may also be associated with small testis, hydrocele, varicocele, and cryptorchidism [11-13], none of which were a presentation of our patient’s balanced translocation. While the importance of AZF genes is well-documented for spermatogenesis, their exact function is not well known. 

The other genetic loci involved in the patient’s translocation are chromosome p32.1, the genetic locus for T-cell acute leukemia protein 1 (TAL1), which codes for a transcription factor involved in the regulation of hematopoiesis and leukemogenesis [14]. While not involved in fertility, translocations that involve this gene have mixed phenotypes. One case report [15] of karyotype t(1;5)(p32;q31) shows no abnormal expression of TAL1, while another study [16] showed two cases of t(1;14)(p32;q11) resulting in T-cell acute lymphoblastic leukemia. This patient’s karyotype and presentation of Y;1, with no known cancer, suggest no aberrant activation of TAL1 when translocated into the Y chromosome.

TESA was performed due to concerns about insufficient sperm concentration for ICSI. Based on clinical experience, we have observed improved outcomes with TESA when sperm is successfully identified in cases of cryptozoospermia, such as in our patient. However, we acknowledge the possibility that no sperm may be recovered during the procedure, which was unfortunately the case with our patient. It is still important to consider TESA as a viable option for cryptozoospermic patients, although studies show decreased chances of successful retrieval compared to micro-TESE [8,17]. However, regional procedural variations can produce comparable tissue and sperm retrieval in TESA as compared to TESE.

Although this case report offers new insight into the implications for patients with cryptozoospermia, further research is needed to identify best practices for the cryptozoospermic male. Male infertility is often multifactorial, which can complicate treatment decisions. In our patient’s case, sperm extraction was initially attempted via TESA. One study found similar sperm retrieval rates between TESA and micro-TESE in patients with severe oligozoospermia; however, among cryptozoospermic patients, micro-TESE demonstrated superior outcomes [17]. Another study showed for cryptozoospermic patients a 73.8% successful live birth rate following intracytoplasmic injection of frozen sperm ejaculate, as well as fresh sperm ejaculated on the day of egg retrieval [18]. Therefore, surgical sperm retrieval may be entirely avoidable in cryptozoospermic patients through the use of ejaculated sperm, an approach ultimately employed in our case following unsuccessful TESA. In cases of NOA, micro-TESE has become the preferred method for sperm retrieval, excising 70-fold less tissue and achieving 1.5 times higher retrieval rates compared to conventional TESE [8,16,19]. However, for cryptozoospermia, the optimal approach, whether surgical retrieval or reliance on ejaculated sperm, appears to be patient-specific. Given the limited fertility insurance coverage across much of the United States, the decision to pursue surgical sperm retrieval, such as micro-TESE, is often challenging. The procedure is significantly more expensive than alternative options and can impose a considerable financial burden on couples [20].

## Conclusions

Causes of male infertility are highly heterogeneous, especially due to the complex nature of the various genetic causes. Balanced Y;1 translocations are not well characterized in the literature, and there is no known treatment to improve reproductive success. While treatments for low sperm count exist and allow high success rates for fertility, there is no standard best practice for cryptozoospermic patients, as treatment is highly patient-dependent and variable.

## References

[1] Stouffs K, Seneca S, Lissens W (2014). Genetic causes of male infertility. Ann Endocrinol (Paris).

[2] Krausz C, Riera-Escamilla A (2018). Genetics of male infertility. Nat Rev Urol.

[3] Braun-Falco M, Schempp W, Nevinny-Stickel-Hinzpeter C, Köhn FM (2007). Azoospermia due to a unique de novo balanced reciprocal translocation (Y;1) (q12;q25). J Androl.

[4] Pabst B, Glaubitz R, Schalk T, Schneider U, Schulze W, Miller K (2002). Reciprocal translocation between y chromosome long arm euchromatin and the short arm of chromosome 1. Ann Genet.

[5] Moreau N, Teyssier M, Rollet J (1987). A new case of (Y;1) balanced reciprocal translocation in an infertile man with Hodgkin's disease. J Med Genet.

[6] Li G, Iqbal F, Wang L (2017). Meiotic defects and decreased expression of genes located around the chromosomal breakpoint in the testis of a patient with a novel 46,X,t(Y;1)(p11.3;p31) translocation. Int J Mol Med.

[7] Hiraki Y, Fujita H, Yamamori S (2006). Mild craniosynostosis with 1p36.3 trisomy and 1p36.3 deletion syndrome caused by familial translocation t(Y;1). Am J Med Genet A.

[8] Alkandari MH, Moryousef J, Phillips S, Zini A (2021). Testicular sperm aspiration (TESA) or microdissection testicular sperm extraction (micro-tese): which approach is better in men with cryptozoospermia and severe oligozoospermia?. Urology.

[9] Brannigan RE, Hermanson L, Kaczmarek J, Kim SK, Kirkby E, Tanrikut C (2024). Updates to male infertility: AUA/ASRM Guideline (2024). J Urol.

[10] (2025). Test menu. https://www.labcorp.com/test-menu/search.

[11] Sun F, Oliver-Bonet M, Turek PJ, Ko E, Martin RH (2005). Meiotic studies in an azoospermic human translocation (Y;1) carrier. Mol Hum Reprod.

[12] Dada R, Gupta NP, Kucheria K (2004). Yq microdeletions-azoospermia factor candidate genes and spermatogenic arrest. J Biomol Tech.

[13] Krausz C, Quintana-Murci L, Barbaux S (1999). A high frequency of Y chromosome deletions in males with nonidiopathic infertility. J Clin Endocrinol Metab.

[14] Vagapova ER, Spirin PV, Lebedev TD, Prassolov VS (2018). The role of TAL1 in hematopoiesis and leukemogenesis. Acta Naturae.

[15] Cho HS, Kim MK, Bae YK (2009). A novel translocation t(1;5)(p32;q31) that was not associated with the TAL1 rearrangement in a case of T lymphoblastic leukemia/lymphoma. Korean J Lab Med.

[16] Bernard O, Barin C, Charrin C, Mathieu-Mahul D, Berger R (1993). Characterization of translocation t(1;14)(p32;q11) in a T and in a B acute leukemia. Leukemia.

[17] Flannigan R, Bach PV, Schlegel PN (2017). Microdissection testicular sperm extraction. Transl Androl Urol.

[18] Hibi H, Tokoro M, Sonohara M, Ihara K, Fukunaga N, Asada Y (2023). Cryptozoospermia: should we use ejaculated sperm or surgically retrieved sperm for assisted reproductive technology?. Reprod Med Biol.

[19] Ghalayini IF, Alazab R, Halalsheh O, Al-Mohtaseb AH, Al-Ghazo MA (2022). Repeated microdissection testicular sperm extraction in patients with non-obstructive azoospermia: outcome and predictive factors. Arab J Urol.

[20] Han TX, Berk B, Ghayda RA, Ernandez J, Kathrins M (2024). Financial decision analysis based on "willingness to pay" for surgical sperm retrieval approaches among men with non-obstructive azoospermia in the United States. Andrology.

